# Retrospective analysis of efficacy, safety, and prognostic factors in a cohort of Chinese hepatocellular carcinoma patients treated with drug-eluting bead transarterial chemoembolization

**DOI:** 10.1590/1414-431X20198467

**Published:** 2019-11-28

**Authors:** Sihan Chen, Rengbin Ji, Xiaojun Shi, Zhe Wang, Dedong Zhu

**Affiliations:** 1 Department of Liver Cancer, Ningbo No. 2 Hospital, Ningbo, China; 2 Department of Cirrhosis, Ningbo No. 2 Hospital, Ningbo, China

**Keywords:** Hepatocellular carcinoma, Drug-eluting bead transarterial chemoembolization, China, Treatment response, Survival, Adverse events

## Abstract

The aim of our study was to assess the efficacy, safety, and prognostic factors of drug-eluting bead transarterial chemoembolization (DEB-TACE) in Chinese hepatocellular carcinoma (HCC) patients. Patients (n=102) diagnosed as primary HCC were consecutively enrolled in this retrospective cohort study. Treatment responses were assessed following the modified Response Evaluation Criteria in Solid Tumors. Progression-free survival (PFS) and overall survival (OS) were evaluated, and adverse events (AEs) as well as liver function-related laboratory indexes of all DEB-TACE records (N=131) were assessed. Complete response (CR) rate, objective response rate, and disease control rate were 51.0, 87.3, and 95.1%, respectively, at 1–3 months post DEB-TACE. The mean PFS and OS were 227 (95%CI: 200–255) days and 343 (95%CI: 309–377) days, respectively. Multivariate logistic regression revealed that portal vein invasion and abnormal total protein (TP) were independent predictive factors for worse CR, and multivariate Cox's regression analysis showed that multifocal disease independently correlated with shorter PFS. Most of the liver function-related laboratory indexes worsened at 1 week but recovered at 1–3 months post-treatment, only the percentage of patients with abnormal ALP increased at 1–3 months. In addition, 112 (85.5%), 84 (64.1%), 53 (40.5%), 40 (30.5%), and 16 (12.2%) patients had pain, fever, nausea, vomiting, and other AEs, respectively. DEB-TACE is efficient and safe in Chinese HCC patients, and portal vein invasion, abnormal TP level as well as multifocal disease could be used as unfavorable prognostic factors to DEB-TACE treatment.

## Introduction

Hepatocellular carcinoma (HCC), the most frequent carcinoma and a leading cause of cancer-related deaths in males with age below 60 years in China, has poor prognosis despite of decreased incidence rate due to control of risk factors such as hepatitis B virus infection and drinking water containing cyanotoxins (1 [Bibr B02] [Bibr B03]–4). Based on accumulating clinical trials and cohort studies, the prognosis assessment and the determination of treatment for HCC patients is now guided by the Barcelona Clinic Liver Cancer (BCLC) staging system (5). In addition to potential curative therapies, including resections, ablation, and liver transplantation, BCLC staging system indicates that for those patients in intermediate stage, transarterial chemoembolization (TACE) is a standard procedure (5).

Driven by the dilemma of relatively severe systemic toxicity and lack of standardization of technique in conventional TACE (cTACE), TACE using drug-eluting beads (DEB-TACE) was introduced using microbeads with a diameter of 100–1000 μm that provide better delivery of chemotherapeutics and more sustained drug concentration while lower concentration in the circulatory system (6,7). With these technique advances, more studies report improved treatment responses and survival as well as less systemic toxicity (8–10).

As one of the developing countries with a huge disease burden of HCC, China has put enormous efforts in the prevention and treatment of HCC over decades. However, the efficacy and safety of DEB-TACE in Chinese HCC patients are not well investigated and this is necessary due to the diversified prevalence and prognosis of HCC, and drug-eluting bead products from abroad. Therefore, the aim of our study was to assess the efficacy, safety, and prognostic factors of DEB-TACE in Chinese HCC patients.

## Material and Methods

### Participants

One hundred and two patients diagnosed with primary HCC from July 20, 2016 to May 31, 2017 at the Department of Liver Cancer in Ningbo No. 2 Hospital were consecutively enrolled in this retrospective cohort study. Patients with the following features were included: 1) diagnosed as primary HCC according to the criteria of American Association for the Study of the Liver Diseases guidelines; 2) above 18 years of age; and 3) about to receive DEB-TACE on demand. In addition, the exclusion criteria were as follows: 1) severe liver or renal failure; 2) sepsis or uncontrollable infection; 3) ascites; 4) history of liver transplantation; 5) contraindication for angiography, embolization procedure, or artery puncture; and 6) women in pregnancy or lactation period. This study was approved by the Ethical Committee of Ningbo No. 2 Hospital and conducted strictly following the principles of Helsinki. Written informed consents were obtained from all participants.

### Data collection

Comprehensive information of HCC patients was documented, including age, gender, history of hepatitis B (HB), history of hepatitis C, history of alcohol drinking, history of cirrhosis, tumor distribution (multifocal and unifocal), tumor location (left liver, right liver, and bilobar), largest nodule size, portal vein invasion, hepatic vein invasion, ECOG performance status (0, 1, 2, and 3), Child-Pugh stage (A, B, and C), BCLC stage (0, A, B, C, and D), cycles of DEB-TACE treatment (1 cycle and 2 or more cycles), and laboratory indexes consisting of white blood cell (WBC), red blood cell (RBC), absolute neutrophil count (ANC), hemoglobin (Hb), platelet (PLT), albumin (ALB), total protein (TP), total bilirubin (TBIL), total bile acid (TBA), alanine aminotransferase (ALT), aspartate aminotransferase (AST), alkaline phosphatase (ALP), blood creatinine (BCr), blood urea nitrogen (BUN), alpha fetoprotein (AFP), carcino-embryonic antigen (CEA), and carbohydrate antigen199 (CA199).

### Assessment of treatment responses, survival, and adverse events

Treatment responses were evaluated by image examination following the modified Response Evaluation Criteria in Solid Tumors (mRECIST) as follows (11): 1) complete response (CR): loss of all arterial enhancement nodules; 2) partial response (PR): equal to or more than 30% decline in the total arterial enhancement nodules; 3) stable disease (SD): nodules that did not meet the criteria of CR or PR, and had an increase in arterial enhancement less than 20%; and 4) progression of disease (PD): an increase of more than 20% in the enhancement nodules or the existence of new nodule formation. Objective response rate (ORR) was the percentage of HCC patients that met the criteria of CR and PR, and disease control rate (DCR) was the proportion of HCC patients that had CR, PR, and SD.

Progression-free survival (PFS) and overall survival (OS) were evaluated. The median follow-up time was 220 days and the last follow-up date was October 20, 2017. Adverse events (AEs) were recorded at 1 month post DEB-TACE, and liver function-related indexes were assessed according to the laboratory findings.

### Drug loading

CalliSpheres^®^ Beads (CBs) (Jiangsu Hengrui Medicine Co, Ltd., China) of 100–300 and 300–500 μm were loaded with 80 mg Epirubicin (Pfizer, USA). The drug loading procedure was as follows: 1) dissolving Epirubicin into solution at 20 mg/mL and storing the solution in a 10 mL syringe; 1) shaking the bottle of CBs and extracting the beads suspension with a 20 mL syringe, standing at room temperature for 5 min; 3) discarding the liquid supernatant, keeping only CBs in the syringe that were mixed with Epirubicin solution by a tee joint; 4) adding non-ionic contrast agent Iopromide (Bayer, Germany) at the ratio of 1:1, and letting the mixture stand for 30 min at room temperature for further application.

### DEB-TACE operation

Each HCC patient underwent DEB-TACE on demand according to assessment of the multi-disciplinary team in our hospital. Firstly, digital subtraction angiography was carried out to detect the tumor’s vascular supply, after the location of which, the hepatic artery was catheterized by a 2.4 F microcatheter (Merit Maestro, Merit Medical System, Inc., USA) using a microwire as the guide by the Seldinger's method. In addition, superselective catheterization (segment/sub segment) was used. Second, CBs loaded with Epirubicin mixed with non-ionic contrast agent were pulsed-injected at the speed of 1 mL/min through the microcatheter into the tumor-supplying artery and stopped when the flow of the contrast agent was static. Another angiography was performed to detect the blushed/tinted tumor after 5 min of the delivery, and the embolization was stopped when there was no more blushed/tinted tumor.

### Statistical analysis

Statistical analysis was performed using SPSS 22.0 software (IBM, USA) and Graphpad Prism 5.01 software (GraphPad Software Inc., USA). Data are reported as means±SD, count (%), or median (25–75th). Comparison between two groups was determined by *t*-test, chi-squared test, or Wilcoxon rank sum test. Kaplan-Meier curves and log-rank test were performed to evaluate the PFS and OS. Univariate and multivariate logistic regressions were conducted to assess the predicting factors for treatment responses, and univariate as well as multivariate Cox's regression analyses were carried out for evaluating the predictive factors for survival data. P<0.05 was considered significant.

## Results

### Characteristics of HCC patients

As reported in Supplementary Table S1, the mean age of the 102 HCC patients was 59.05±11.46 years, among whom there were 18 females and 84 males. Thirty-seven (36.3%) patients had multifocal tumors and 65 (63.7%) had unifocal tumors. Tumors were located in the left liver in 15 (14.7%) patients and in the right liver in 64 (62.8%) patients, and the remaining 23 (22.5%) patients had bilobar disease. The median value of the largest nodule size was 3.30 (2.18–7.03) cm, and the number of patients with portal vein invasion and hepatic vein invasion were 25 (24.5%) and 5 (4.9%), respectively. In addition, the numbers of patients in BCLC stage 0, A, B, C, and D were 2 (2.0%), 29 (28.4%), 32 (31.4%), 31 (30.4%), and 2 (2.0%), however, in 6 (5.8%) patients, the information of BCLC stages could not be assessed. As for the number of DEB-TACE cycles of patients, 73 (71.6%) patients received 1 cycle and 29 (28.4%) patients received 2 cycles. Moreover, there were 7 (6.9%) patients who had surgery, 9 (8.8%) who received radiofrequency ablation, 4 (3.9%) who were treated by alcohol injection, and 2 (2.0%) who received apatinib treatment post DEB-TACE treatment. Other information of clinical history, staging, and liver functions as well as the laboratory indexes are shown in Supplementary Table S1.

### Treatment responses according to mRECIST

The treatment responses were evaluated at 1–3 months after DEB-TACE procedures by image examinations, showing that ORR was 87.3% and the DCR was 95.1% (Table 1).

**Table 1:** Treatment response by drug-eluting beads transarterial chemoembolization.

Treatment response	Patients (n=102)
Complete response	52 (51.0)
Partial response	37 (36.3)
Stable disease	8 (7.8)
Progressive disease	3 (2.9)
Not assessed	2 (2.0)
Objective response rate	89 (87.3)
Disease control rate	97 (95.1)

Data are reported as count (percentage).

### PFS and OS

As displayed in Figure 1, the mean PFS was 227 (95%CI: 200–255) days and the mean OS was 343 (95%CI: 309–377) days in HCC patients post DEB-TACE.

**Figure 1:** Progression-free survival (PFS) and overall survival (OS) in hepatocellular carcinoma patients treated by drug-eluting bead transarterial chemoembolization. Kaplan-Meier curve and log-rank test were used. P<0.05 was considered significant.

### Analyses of factors affecting CR and ORR

As presented in Supplementary Table S2, univariate logistic regression showed that multifocal disease (P=0.002), bilobar tumor location (P=0.011), largest nodule size >3.3 cm (P<0.001), portal vein invasion (P<0.001), higher ECOG performance status (P<0.001), higher BCLC stage (P=<0.001), abnormal ALP (P=0.025), and abnormal AFP (P=0.001) were factors for predicting worse CR. Factors with a P value <0.1 were included in the multivariate logistic regression, and portal vein invasion (P=0.003) as well as abnormal TP (P=0.025) were found to be independent predictive factors for unfavorable CR.

Univariate logistic regression revealed that portal vein invasion (P=0.019), higher ECOG performance status (P=0.027), and higher BCLC stage (P=0.018) were negatively correlated with ORR. All factors with a P value <0.1 were included in the multivariate logistic regression, which displayed that no factor was an independent predictive factor for ORR (Supplementary Table S3).

### Analyses of factors for predicting survival

To analyze the predictive value of baseline characteristics for PFS, univariate and multivariate Cox's regression analyses were performed, showing that multifocal disease (P<0.001), bilobar tumor location (P=0.001), largest nodule size >3.3 cm (P=0.002), portal vein invasion (P<0.001), hepatic vein invasion (P<0.001), higher ECOG performance status (P<0.001), higher BCLC stage (P<0.001), combination of ordinary embolization agent (P=0.024), and abnormal AFP (P=0.001) were negatively associated with PFS (Supplementary Table S4). Multivariate analysis revealed that only multifocal disease (P=0.050) was an independent predictive factor for worse PFS. As listed in Supplementary Table S5, multifocal disease (P=0.002), bilobar tumor location (P=0.001), largest nodule size >3.3 cm (P=0.003), portal vein invasion (P<0.001), higher ECOG performance status (P<0.001), higher BCLC stage (P<0.001), RBC abnormal (P=0.025), abnormal ALB (P=0.025), abnormal TBA (P=0.024), abnormal ALP (P=0.009), abnormal AFP (P=0.003), and abnormal CEA (P=0.004) were factors for predicting worse OS. However, a history of HB (P=0. 046) and tumor location on right liver (P=0.046) predicted better OS. All factors with a P value <0.1 were included in multivariate Cox's regression analysis, which demonstrated that there was no independent predictive factor for OS.

### Liver function

Laboratory indexes were recorded for the evaluation of liver function change prior to and after each DEB-TACE record (N=131). As presented in Table 2, the percentage of patients with abnormal ALB (P<0.001), abnormal TP (P<0.001), abnormal ALT (P<0.001), and abnormal AST (P=0.002) increased at 1 week but were not different compared to baseline (P=1.000, P=1.000, P=0.307, and P=0.557, respectively) post DEB-TACE. However, the proportion of patients with abnormal ALP was similar to baseline at 1 week (P=0.125) but was notably elevated at 1–3 months (P=0.001). In addition, the number of patients with abnormal TBIL (P=0.134 and P=0.401) and abnormal TBA (P=1.000 and P=1.000) did not change at both 1 week and 1–3 months post DEB-TACE.

**Table 2:** Liver function before and after drug-eluting bead transarterial chemoembolization (DEB-TACE) treatment in hepatocellular carcinoma patients (131 records).

Count (n/N/%)	Baseline	1 week post DEB-TACE	1–3 months post DEB-TACE	P value*	P value^#^
ALB abnormal	75/130 (58)	110/128 (86)	76/117 (65)	**<0.001**	1.000
TP abnormal	30/130 (23)	66/127 (52)	31/117 (27)	**<0.001**	1.000
TBIL abnormal	35/130 (27)	46/128 (36)	41/117 (35)	0.134	0.401
TBA abnormal	60/129 (47)	59/121 (49)	62/115 (54)	1.000	1.000
ALT abnormal	18/130 (14)	52/128 (41)	23/117 (20)	**<0.001**	0.307
AST abnormal	51/130 (39)	62/128 (48)	54/117 (46)	**0.002**	0.557
ALP abnormal	54/129 (42)	49/122 (40)	65/114 (57)	0.125	**0.001**

Analysis was based on 131 DEB-TACE records. Comparison was determined by the McNemar test. Bold type indicates statistical significance. *P<0.05 between indexes from baseline to 1 week post-treatment. ^#^P<0.05 between indexes from baseline to 1–3 months post-treatment. ALB: albumin; TP: total protein; TBIL: total bilirubin; TBA: total bile acid; ALT: alanine aminotransferase; AST: aspartate aminotransferase; ALP: alkaline phosphatase.

### AEs post DEB-TACE

AEs were recorded according to each DEB-TACE record (N=131). The majority of records reported fever (112 (85.5%)) at 1 week post DEB-TACE (Table 3).

**Table 3:** Adverse events one week after drug-eluting bead transarterial chemoembolization treatment in hepatocellular carcinoma patients (131 records).

Adverse events	n (%)
Fever	112 (85.5)
Pain	84 (64.1)
Nausea	53 (40.5)
Vomiting	40 (30.5)
Others	16 (12.2)

## Discussion

The results in our study showed that: 1) CR, ORR, and DCR at 1–3 months post DEB-TACE were 51.0, 87.3, and 95.1%, respectively; 2) the mean values of PFS and OS were 227 days and 343 days; 3) multivariate logistic regression revealed that portal vein invasion and abnormal TP predicted unfavorable CR independently, and multivariate Cox's regression analysis displayed that multifocal disease was an independent predictive factor for shorter PFS; and 4) the percentage of patients with abnormal ALP did not change at 1 week but increased at 1–3 months post DEB-TACE, and the most common AEs were fever and pain after DEB-TACE.

Slow release of chemotherapeutics and a higher drug concentration in tumor tissue make it possible for physicians to achieve a better ischemic and cytotoxic impact on the tumor through DEB-TACE (7). The microbeads are essential for accomplishing this, and there are multiple available microbeads. The beads used in our study were Callispheres^®^ beads, the first chemoembolization product in China. A previous *in vitro* experiment showed that compared with lipiodol infusion, CBs deliver a higher dose of doxorubicin within the area of 200 μm from the bead edge and could last for over 1 month in rabbits, indicating CBs deliver chemotherapeutics effectively (12). However, clinical studies on CBs in China are rare. In the study of Kloth et al. (13), 28.6, 42.8, and 28.6% of their HCC patients achieved CR, PR, and SD after DEB-TACE using biphasic contrast-enhanced CT image for treatment response evaluation. Another retrospective cohort study reports an ORR of 94.3% among median stage HCC patients, in which the CR and PR rates were 42.4 and 57.6% (14). In addition to HCC patients in intermediate stage, DEB-TACE has been used in patients with liver metastasis as well. A multicenter prospective, non-controlled clinical trial in the USA illustrates that 55% of patients with liver dominant metastasis from melanoma achieved tumor response (CR+PR) and 80% displayed disease control (CR+PR+SD) after DEB-TACE treatment (15). The treatment response rates vary from study to study. The CR rate in our study was numerically higher and our ORR was numerically lower compared with those previous studies, which might be the result of the diversified patient eligibility, sample size, or the technique used for treatment response assessment. DEB-TACE is reported to be superior to cTACE in improving the survival of HCC patients (16).

In a single-center, single-arm, retrospective cohort study using small size drug-eluting beads for HCC patients, the median OS was 42 (95%CI: 38–43) months post DEB-TACE treatment (17). In another retrospective cohort study, patients with HCC in median stage had a mean PFS of 10.9 months and a mean OS of 33.9 months after DEB-TACE under cone beam computed tomography (14). A study that evaluated the efficacy of DEB-TACE compared with cTACE in HCC patients found that the median time to progression and mean OS in DEB-TACE group were 10.8 and 46.6 months, respectively (18). The survival of HCC patients post DEB-TACE are influenced by multiple factors, including the follow-up time, treatment response, and patient eligibility. The mean value of PFS and OS were numerically shorter in this study than some of the previous studies, which could be caused by the relatively short follow-up time in this study.

Prognostic factors for efficacy of DEB-TACE for HCC patients is rarely investigated. Several prognostic factors have been identified by prior studies; for example, a retrospective cohort study reports that tumor location in the segments I and IV predicts worse CR while tumor size below 5 cm is correlated with better CR, both factors are independent predictive factors (19). The multivariate logistic regression and Cox's regression analysis in our study found that portal vein invasion, abnormal TP, and multifocal disease independently predicted unfavorable efficacy. Portal vein invasion suggests a metastasis of the disease, a phase in which HCC patients with advanced stage can only receive palliative treatment according to BCLC staging system (5). A retrospective study evaluating the efficacy, safety, and prognostic factors of cTACE that used gelatin sponge particle with a diameter of 350-560 μm combined with chemoembolization for HCC patients elucidates that the portal vein invasion is an independent predictive factor for poor survival (20). Abnormal TP, which strongly suggests liver function deterioration, was associated with poor CR in our study. The status of liver function evaluated by Child-Pugh staging is a prognostic factor for efficacy of HCC patients after treatments, including TACE treatment (21,22), which might be a possible explanation for the result in our study. Another independent predictive factor was multifocal disease, which is elucidated to be independently associated with poor survival after TACE, according to previous studies (23).

Operations on patients always cause short-term liver damage. The procedure of DEB-TACE requires hepatic artery puncture and infusion, which impairs the artery and liver tissue temporarily and contributes to abnormalities of liver function-related laboratory indexes. In our study, most indexes deteriorated at 1 week but were better at 1–3 months after DEB-TACE, indicating that liver function experienced temporary damage but recovered chronically. However, the percentage of patients with abnormal ALP increased at 1–3 months despite it being similar to baseline at 1 week post-treatment. Several previous studies found that ALP could independently predict the prognosis of HCC patients undergoing TACE, suggesting ALP might be strongly correlated with prognosis (24,25). Another probable reason might be that ALP also associates with cancer cells proliferation and inflammation of tumor tissue in HCC (26,27). Thus, although the liver function recovered, ALP kept worsening probably because it is correlated with not only the liver function but also the pathological progress of HCC.

DEB-TACE reduces severe complications by eliminating the systemic concentration of chemotherapeutics owing to the utilization of tiny microbeads and superselective catheterization (21,28). Embolization syndrome is common among HCC patients during and after DEB-TACE treatment. In our study, pain and fever were the most frequent AEs, and the proportion of patients with nausea and vomiting were relatively decreased, which are in accordance with most of the previous studies (9,29). Pain is mostly caused by the arterial catheterization and chemoembolization, and fever is primarily due to the inflammatory responses during and post DEB-TACE. Those AEs were very manageable and were properly treated in our hospital.

There were some limitations in our study: 1) as a single center study, there might be selection bias due to all patients being from a local region; 2) the follow-up time of our study was relatively short, which could be prolonged in the future; 3) the data of our patients were retrospectively analyzed, which might cause bias and confounding factors, such as recall bias. Therefore, a prospective, multicenter cohort study with longer follow-up time is needed.

In conclusion, DEB-TACE seemed to be efficient and safe in Chinese HCC patients. Portal vein invasion, abnormal TP level, as well as multifocal disease could be used as unfavorable prognostic factors to DEB-TACE treatment.

## Supplementary Material

Click here to view [pdf].
